# Assessment of composition and spatial dynamics of weed communities in agroecosystem under varying edaphic factors

This article has been retracted.

**DOI:** 10.1371/journal.pone.0266778

**Published:** 2022-05-27

**Authors:** Anum Yousaf, Noreen Khalid, Muhammad Aqeel, Zarrin Fatima Rizvi, Haifa A. S. Alhaithloul, Wajiha Sarfraz, Khalid Al Mutairi, Tasahil S. Albishi, Saad Alamri, Mohamed Hashem, Ali Noman, Sameer H. Qari

**Affiliations:** 1 Department of Botany, Government College Women University, Sialkot, Pakistan; 2 State Key Laboratory of Grassland Agro-Ecosystems, School of Life Sciences, Lanzhou University, Lanzhou, PR China; 3 Biology Department, Collage of Science, Jouf University, Sakaka, Saudi Arabia; 4 Biology Department, Faculty of Science, University of Tabuk, Tabuk, Saudi Arabia; 5 Biology Department, College of Applied Sciences, Umm Al-Qura University, Makkah, Saudi Arabia; 6 Department of Biology, Faculty of Science, King Khalid University, Abha, Saudi Arabia; 7 Botany and Microbiology Department, Faculty of Science, Assiut University, Assiut, Egypt; 8 Department of Botany, Government College University, Faisalabad, Pakistan; 9 Department of Biology, Al-Jumum University College, Umm Al-Qura University, Makkah, Saudi Arabia; Ghazi University, PAKISTAN

## Abstract

Weeds are important components of the agroecosystems due to their role as primary producers within the farming systems, yet they are considered as major constraints to crop production. A phytosociological study was conducted to assess the composition and spatial distribution of existing weed species under the influence of various edaphic factors in the 15 wheat fields. Quadrat method was applied and different phytosociological attributes including abundance, density, and frequency were estimated by randomly laying down 10 square-shaped quadrats of size 1m^2^ in each wheat field. A total of 34 weed species belonging to 17 families and 30 genera were explored from 150 quadrats. Fabaceae and Asteraceae were ubiquitous plant families. Various edaphic factors such as; soil texture, electrical conductivity, soil pH, total dissolved solids, nitrogen, calcium carbonate, organic matter, NaCl, calcium, phosphorous, potassium, sodium, and zinc were determined. Pearson’s correlation was employed to correlate weeds and the potential edaphic variables. The results depicted that most of these weed pairs’ associations correlated positively. Simultaneously, the abundant weed species including *Trifolium repens*, *Coronopus didymus*, and *Urtica dioica* showed a positive correlation with most of the investigated ecological variables.

## Introduction

Wheat (*Triticum aestivum* L.) is an annual, autogamous crop that is grown on an area of about 237 million hectares across the globe, constituting a yield of 749 million tonnes [1]. This crop is a main dietary component for approximately one-third of the total global population. Wheat is acclimated to the latitudes of 30° and 60°N, and 27° and 40°S on the globe. It grows at an optimum temperature of 25° C with precipitation varying between 250 to 1750 millimeters. Practically, 1/6 of the total world’s fertile land is under wheat cultivation, making it a major product in the global food market. It is a mostly-consumed agricultural product in Pakistan cultivated on an area of around 9 million hectares which is roughly 40% of the country’s total fertile land [2].

Weeds as an integral component of a dynamic ecosystem, often emerge as pioneer plants in secondary succession and ultimately expand as an obtrusive participant with food crops [3]. The notion of weed as an undesirable plant was originally realized when humans begin to establish plants for their nutritional benefits. Holm et al., [4], classified 250 substantial weed species for agricultural uses across the world. In agro-ecosystems, weeds have been remained a persisting impediment to crop yield, owing to the ideal features they possess that includes its active transpiration rate, allelopathy, ecological flexibility, effective stomatal conductance, efficient seed dispersal method, fast reproduction rate, higher photosynthetic activity, rapid seed development, short life cycle and higher resilience to ecological stresses [5, 6].

Weeds pose a global threat to crops as their populations vary both spatially and temporally which induce substantial crop damage in arable fields with an estimated yield loss of about 10 to 80% [7, 8]. Weeds are perceived as the most significant adversary of the wheat crop as they induce delays in wheat harvest, reduce its kernel quality, and inflate the operational expenses for cleaning and threshing. Globally, the reduction in wheat yield brought about by the weeds is approximated to be 13.1% [9]. In Pakistan, the rampant growth of weeds causes an estimated yield loss of 20 to 40% of the wheat crop adding up to more than 28 billion rupees at the national scale [10].

Weeds compete with crops for limited natural resources such as minerals, light, and dampness. Moreover, they are highly adaptable to new weed control and management strategies. The variations in the spatial pattern of weeds mainly depend on various anthropogenic and ecological factors such as no-tillage practices, herbicide application, and crop rotation which cause significant variations in weed densities [11, 12]. Rew and Cousens [13], observed that a site-specific weed species composition related to spatial soil heterogeneity often occurs within arable fields. Various soil properties including soil organic carbon, nutrient status of the soil, and soil texture primarily influence weed growth and its composition in a rather complex way, therefore, one must consider different inter-relations [6, 14].

Currently, various advanced approaches are being employed to accurately predict weed occurrence in the fields. But until now, the precise weed data correlated to various soil properties is limited, even though soil sensing approaches ensure soil data evaluations at high spatial resolution. Variability in the weed community structure and its distribution is chiefly influenced by various ecological drivers including crop type and its sustainability, farm management practices, physico-chemistry of the soil, seasonality, and urbanization [15].

The scope of the current investigation was to document and correlate weed data with soil properties to determine the influence of edaphic variants on the composition and spatial distribution of weed species of wheat crop of Sialkot, Pakistan. A prerequisite for the research was to employ a multivariate statistical approach that would further aid in developing a sustainable interminable plan for effective weed control management.

## Materials and methods

### Study area

The current research was conducted during the Rabbi season (December 2019 –April 2020) to investigate the weed ecology of 15 different fields of Sialkot, where the wheat crop has sporadically been cultivated. Sialkot is situated at an altitude of 256 meters above sea level, between 32°30’ North latitude and 74°31’ East longitude, in the North-East of the Punjab Province, Pakistan (Fig 1). It features a humid subtropical climate and expands on an area of around 1900 hectares which comprises about 637 villages. Approximately, 169.32 acres (4.2%) of Sialkot’s total land is utilized for agriculture purposes. The grains were sown during late November 2019, followed by the irrigation and plowing of the fields which were frequently visited to explore the weed flora. The quantitative ecological approach i.e., the quadrat method was applied after Clements [16]. And phytosociological attributes such as density, frequency, and abundance of weed species were estimated by establishing 10 square-shaped quadrats on each of the 15 wheat fields (a total of 150 quadrats) having a size of 1m^2^ in each projected area. Sub-tropical deciduous vegetation such as *Acacia nilotica*, *Albizzia lebbek*, *Azadirachta indica*, *Bombax ceiba*, *Cassia fistula*, *Dalbergia sissoo*, *Eucalyptus camaldulensis*, *Melia azedarach*, *Morus alba*, *Pongamia pinata*, *and Vaccinium myrtillus* inhabited the land. Furthermore, herbicides are seldom sprayed by native farmers, hence weeds are thriving abundantly.

**Fig 1:** Study area along with sites in district Sialkot, Pakistan.

### Weed identification

Weed species were identified by reviewing accessible literature [17–22].

### Phytosociological attributes

Community attributes such as abundance, density and frequency of each weed species were recorded following Odum [23].


$$Abundance=\frac{Total\;number\;of\;weed\;species\;in\;all\;quadrats}{Total\;number\;of\;quadrats\;in\;which\;individual\;species\;occur}$$

$$\%\;Density\;\left(D\right)=\frac{Total\;number\;of\;individual\;species\;in\;all\;quadrats}{Total\;number\;of\;quadrats}\;\text{x}\;100$$

$$\%\;Frequency\;\left(F\right)=\frac{Number\;of\;quadrats\;in\;which\;a\;weed\;species\;occurred}{Total\;number\;of\;quadrats}\;\text{x}\;100$$

Acquired data was put in a tabulated form to correlate it with the soil properties of the investigated area.

### Soil sampling

Three soil samples (a total of 45 samples) were collected at 15cm to 20cm depths from each of the 15 wheat fields during the survey conducted in 2019–2020 during the Rabbi season. In each field, 3 random areas were marked and dug with a blunt knife to retrieve 500g of soil. Each soil sample was put in a polythene bag accompanying a tag on which sample number, date and place of the collection were specified. A set of 45 soil samples were then brought to the laboratory for further analysis to discover the inherent fertility and textural class of the observed soil.

During physico-chemical analysis, various parameters including calcium carbonate, concentration of Ca^+^, K^+^, Na^+^, P^+^, Zn and total nitrogen, electrical conductivity (EC), NaCl%, organic matter, soil pH, total dissolved solids (TDS), and texture were recorded using conventional laboratory techniques. A flame photometer (Flame photometer 410, Corning) was used to record K^+^ and Na^+^ ions whereas, an Atomic Absorption Spectrophotometer (Perkin Elmer Analyst 100) was utilized to determine the concentrations of Ca^+2^, P, Zn and N in the observed soil samples. Soil texture was demonstrated by the feel method. To determine the lime content of these soil samples, acid neutralization method was employed. Approximately, 5g of soil was initially treated with 0.5N hydrochloric acid and then titrated with 0.025N sodium hydroxide while using phenolphthalein as an acid-base indicator. Meanwhile, the standard sequential LOI (Loss on ignition) method was applied for soil OM (organic matter) measurement [24]. The investigated samples were air dried and mixed homogeneously followed by grounding. 2g of each pulverized sample was passed through a 60 μm mesh. These samples were later measured in 20 ml crucibles and were placed overnight inside an oven at 105°C. Subsequently, cooled in desiccators, the air-dried samples were again weighed to find the residual moisture content. Loss on ignition of the organic matter was estimated by the equation:

$$Loss\;on\;ignition\;at\;105{}^{\circ}C=\frac{100(weight\;of\;the\;air\;dried\;sample-\;Dry\;weight\;of\;the\;sample\;heated\;at\;105{}^{\circ}C)}{Weight\;of\;the\;air\;dried\;sample}$$

In a flask, 25g of each sample was taken and supplemented up to 100ml by distilled water for demonstrating the soil pH, TDS, EC and NaCl%. The mixture was stirred by manual shaking for about 10 minutes straight and then was properly stirred for 6 hours on a shaking machine in order to segregate the suspended matter from the solution. A Whatman filter paper No.1 was used to filter the aforementioned solution. Afterwards, soil pH, NaCl% and EC were measured by pH meter and conductivity meter, respectively [25]. While, soil TDS was recorded by TDS meter (Hanna HI 83141).

### Data analysis

Multivariate ordination techniques are successfully applied in soil-plant research to analyze multi-dimensional data viz., edaphic factors and population [26]. The collective data of 150 quadrats was organized in MS excel and PC-ORD version 5 was adopted to perform Principal Component Analysis (PCA) in order to demonstrate the influence of various edaphic factors on spatial heterogeneity of weed species [27]. Ordination diagrams (attribute biplots) were derived through Canoco version 4.5 to display the relationship between weed communities of the observed localities and various attributes. Also, Pearson Correlation was used to correlate different weed species as well as with other ecological variables. Pearson correlation is a linear correlation, where positive correlation suggests that two weed species representing mutualism or weak parasitism and have similar requirements for environmental factors are likely to emerge simultaneously. Whereas, a negative correlation indicates the exclusive appearance of two weed species in the plots primarily on account of definite ecological requirements, interference and competition among them. Species richness, Shannon index of α-diversity, and species evenness were carried out to identify similarity. While, Non-metric multidimensional scaling (NMDS) based on Bray-Curtis dissimilarity matrices, including analysis of similarity (ANOSIM) was carried out to test dissimilarity among existing weed species at different sites.

## Results

### Density (m^-2^)

The recorded weed data exhibits that 34 weed species were documented in 15 wheat fields of Sialkot, Pakistan (Fig 2). Salehpur (80.5), Ajuwali (70.3), and Kala Khambra (65.7) were identified as the most intensely weed infested locations, whereas the weed density was relatively low in Pindi Panjoran (13). The investigated area of Sialkot was mostly dominated by *Trifolium repens* (108.4), *Coronopus didymus* (83.6) along with *Urtica dioica* (73.3) and *Anagallis arvensis* (70). Meanwhile, *Portulaca oleraceae* (0.7), *Oxalis corniculata* (0.6) and *Malva parviflora* (0.4) emerged as minor weeds in only one or two locations of studied area.

**Fig 2:** Chord diagram representing the density of recorded weed species in fifteen different wheat fields of Sialkot.

After the weed community composition data were transformed for chord distance, the relationship between densities of weed communities from various wheat fields was then explored via principal component analysis (PCA). Most weed assemblages in the wheat fields of Khambranwala, Salehpur, and Kapurowaali were characterized by positive values along the PC1 (first principal component). The weed associations in the aforementioned fields were significantly different from rest of the wheat fields as evident in the PCA biplot (Fig 3). Overall, all 34 weed species contributed strongly to the first two principal components as displayed by the labelled vectors (Fig 3). Twenty one (21 out of 34) of the weed species contributed to a larger %age in Khambranwala, Salehpur and Kapurowaali wheat fields whereas 13 (13 out of 34) of them were relatively more abundant in the rest of the wheat fields in Sialkot.

**Fig 3:** PCA biplot for analyzing relationship between weed communities’ density in different wheat fields.

Principal component analysis was performed for analyzing weed frequency from fifteen surveyed wheat fields in Sialkot. First principal component axis was mostly represented by 19 (19 out of 34) weed species of Khambranwala, Ajuwali, Salehpur, Sagarpur, and Kapurowaali while the remaining 15 (15 out of 34) of them represent the rest of the wheat fields. The weed species were relatively more frequent in Ajuwali as denoted by labelled vectors in first principal component of the PCA biplot. *T*. *repens* was the most frequent weed species as shown in the PCA biplot. *Melilotus indicus* was mostly associated with Salehpur fields (Fig 4).

**Fig 4:** PCA biplot for analyzing relationship between weed communities’ frequency in different wheat fields.

### Correlation among different weed species

Correlation data (Fig 5) on different weed species indicates that at 99% confidence level, *Cynodon dactylon-T*. *repens* and *M*. *indicus-T*. *repens* correlate strongly negative with each other. Meanwhile, weed species pairs: *A*. *arvensis-E*. *helioscopia*, *Centella asiatica-Sonchus oleraceus*, *C*. *arvense-O*. *corniculata*, *C*. *arvense-Parthenium hysterophorus*, *C*. *arvense-Plantago lanceolata*, *Convolvulus arvensis-Lathyrus aphaca*, *C*. *arvensis-Medicago polymorpha*, *C*. *arvensis-P*. *repense*, *L*. *aphaca-P*. *repense*, *M*. *polymorpha-P*. *repense*, *O*. *corniculata-P*. *hysterophorus*, *O*. *corniculata-P*. *lanceolata*, and *P*. *hysterophorus-P*. *lanceolata* show a strong positive correlation.

**Fig 5:** Correlation matrix of different weed species. Asterisk (*) sign denotes significant relationship (p ≤ 0.05).

Furthermore, moderately positive correlated weed species are: *A*. *arvensis-M*. *denticulata*, *A*. *arvensis-Melilotus alba*, *B*. *napus-M*. *polymorpha*, *B*. *napus-M*. *indicus*, *C*. *sativa-R*. *obtusifolius*, *C*. *sativa-S*. *oleraceus*, *C*. *asiatica-C*. *album*, *C*. *arvense-M*. *indicus*, *C*. *arvense-P*. *plebeium*, *C*. *arvense-R*. *obtusifolius*, *C*. *arvensis-Glechoma hyderaceae*, *C*. *arvensis-V*. *sativa*, *C*. *didymus-P*. *oleraceae*, *C*. *dactylon-M*. *indicus*, *C*. *dactylon-P*. *plebeium*, *Digitaria sanguinallis-Festuca rubra*, *E*. *helioscopia-M*. *polymorpha*, *E*. *helioscopia-P*. *repense*, *G*. *hyderaceae-L*. *aphaca*, *G*. *hyderaceae-M*. *polymorpha*, *G*. *hyderaceae-P*. *repense*, *G*. *hyderaceae-V*. *sativa*, *L*. *aphaca-M*. *polymorpha*, *M*. *denticulata-M*. *alba*, *M*. *polymorpha-M*. *indicus*, *M*. *polymorpha-V*. *sativa*, *M*. *indicus-P*. *plebeium*, *O*. *corniculata-P*. *plebeium*, *O*. *corniculata-R*. *obtusifolius*, *P*. *repense-V*. *sativa*, *P*. *hysterophorus-P*. *plebeium*, *P*. *hysterophorus-R*. *obtusifolius*, *P*. *lanceolata-P*. *plebeium*, *P*. *lanceolata-R*. *obtusifolius*, *P*. *plebeium-R*. *obtusifolius* and *R*. *dentatus-S*. *marianum*.

### Correlation among different edaphic factors

A correlation analysis of the data of different edaphic factors demonstrates some significant negative and positive relations among them (Fig 6). EC and TDS show significant positive correlation with each other. Whereas, Zn has shown a significant negative correlation with N. Other than this, we could not find a strong positive or strong negative correlation among edaphic factors generally.

**Fig 6:** Correlation among various edaphic factors. Abbreviations used are TDS (total dissolved solids); OM (organic matter); EC (electrical conductivity).

### Correlation between weed species and different edaphic factors

Composition and distribution of different weed species varies spatially due to the influence of various edaphic variables. Pearson correlation data on different edaphic factors and weed species demonstrates the positive and negative relationship between them (Fig 7). It was indicated that pH correlates negatively with *S*. *oleraceus*, *C*. *album*, and *C*. *asiatica*, while it correlates positively with *M*. *polymorpha* and *C*. *arvensis*. Whereas, TDS shows a negative correlation with *M*. *indicus* and *C*. *dactylon* and positive correlation with *T*. *repens*, *P*. *oleraceae*, and *C*. *asiatica*. EC, K, and Ca correlate positively with *C*. *asiatica*, *M*. *parviflora*, and *C*. *sativa*, respectively. Na shows a negative relationship with *D*. *sanguinallis* and *C*. *sativa*, simultaneously, P correlates negatively with *M*. *alba*, *M*. *denticulata*, *E*. *helioscopia*, and *A*. *arvensis*. It was also observed that Zn showed a positive correlation with *M*. *neglecta*. Meanwhile, CaCO_3_ correlates positively with *R*. *dentatus* and negatively with *P*. *plebeium*, *M*. *indicus*, and *C*. *dactylon*. Furthermore, NaCl correlates positively with *L*. *aphaca*, *D*. *sanguinallis*, and *C*. *arvensis* and nitrogen correlates negatively with *M*. *neglecta*.

**Fig 7:** Correlation data on weed species and different edaphic factors. Abbreviations used are TDS (total dissolved solids); OM (organic matter); EC (electrical conductivity). * denotes significant interaction at p ≤ 0.05, and ** denotes significant interaction at p ≤ 0.01.

### Relative abundance

The weed species abundance data (Fig 8) displayed that wheat fields of Salehpur, Ajuwali, Kapurowaali, Sagarpur, and Khambranwala exhibited highest abundance of different weed species. While, Bhagwal Awanan site showed fewer number of respective weed species compared to other fields. *T*. *repens* was the most abundant weed species that was found abundantly in ten out of fifteen wheat fields followed by *C*. *didymus* (9 fields) and *U*. *dioica* (5 fields). On the other hand, *O*. *corniculata*, *P*. *repense* and *M*. *parviflora* were rare weed species that were present in only one or two of the 15 investigated wheat fields.

**Fig 8:** Relative abundance of 34 weed species in 15 different wheat fields of Sialkot.

### Diversity indices

According to Shannon index, the α-diversity of plant species found to be greatest at Ajuwali, followed by Salehpur and Sagarpur sites (Fig 9a). Of all the sites studied, the median value of α- diversity was noted at Ballanwala. However, the lowest α-diversity based on Shannon’s index, was recorded at Saidpur site. Taking into consideration the species richness and evenness, Kapurowaali site had the highest species evenness (Fig 9b), species richness was, however, found to be highest at Ajuwali (Fig 9c).

**Fig 9:** Alpha diversity (Shannon index) (a), Species evenness (b), and species richness (c) of weeds at various study sites. * shows significance at p ≤ 0.05, ** shows significance at p ≤ 0.01, *** indicate significance at p ≤ 0.001, and **** indicate significance at p ≤ 0.0001.

Moreover, NMDS ordination, based on Bray-Curtis dissimilarity matrices, explained significantly (ANOSIM, R = -0.301, P = 0.7593, Stress = 0171265) distinct variation among different sites. Beta-diversity using NMDS ordination revealed that weed communities in studied sites had different pattern, and provided distinct clustering of weed communities related to sites (Fig 10).

**Fig 10:** Non-metric multidimensional scaling (NMDS) based on Bray-Curtis dissimilarity matrices showing beta-diversity among different studied sites. AW: Ajuwali; BA: Bhagwal Awanan; BW: Ballanwala; CM: Chak Mandhaar; JK: Jorian Kalan; KB: Kotli Bhutta; KK: Kala Khambra; KP: Kapurowaali; KW: Khambranwala; LP: Lalpur; MK: Machi Khokhar; PP: Pindi Panjoran; SG: Sagarpur; SL: Salehpur; SP: Saidpur.

## Discussion

The present investigation is demonstrated on the culmination of the survey carried out in wheat fields of Sialkot, Punjab, Pakistan. The survey was conducted during winter season (December 2019 to April 2020) to appraise the floristic spectrum of weed species in wheat crops of Sialkot. The current research established 34 weed species belonging to 17 families and 30 genera assorted in about 150 quadrats. About 30 of them (88.23%) were dicotyledonous whereas the rest of 4 weed species (11.76%) were monocotyledonous. The eudicot families; Fabaceae (7 weed species) and Asteraceae (5 weed species) were the predominant lineages of the 17 families recorded in the research area, followed by the monocot family Poaceae (4 weed species) and eudicot family Polygonaceae (3 weed species).

In terms of weed species richness, the order of families found in Sialkot region was as follow: Fabaceae, Asteraceae, Poaceae, Polygonaceae, Brassicaceae, Malvaceae, Amaranthaceae, Apiaceae, Cannabaceae, Convolvulaceae, Euphorbiaceae, Lamiaceae, Oxalidaceae, Plantaginaceae, Portulaceae, Primulaceae and Urticaceae. Khattak et al., [28] reported a total of 43 weed species associated with 17 families. Among them, Asteraceae was the predominant family which was also observed in the current investigation. Poaceae was also reported as the most prominent weed family in the PMAS Arid Agriculture University, Rawalpindi campus during a survey supervised from 2007 to 2008 [29]. The current study also complies with the works of [30–33], who also recorded Fabaceae and Poaceae as the most substantial families.

The floristic spectrum of surveyed fields also depicts that the wheat crop has its suite of selective weed species [8, 34]. The current findings also reciprocate the works of Hyvönen et al., [11] and Marwat et al., [8] who observed the higher number of weeds species particularly dicotyledonous species in wheat fields mainly due to cultivation inputs inadequacy. The most predominant weed species in the studied fields were *T*. *repens*, *C*. *didymus* along with *U*. *dioica* and *A*. *arvensis*. Gupta et al., [35] recorded *A*. *arvensis* and *C*. *album* as the most abundant weeds species that actively compete with wheat crop for light, space, and moisture.

Physico-chemical properties of soil, crop rotation, and diverse farming practices greatly affects the diversity and richness of weed species [13]. Weed composition data on the wheat fields of Sialkot disclosed that the estimated densities and spatial patterns of studied weed species were distributed heterogeneously throughout the region. Ritter and Gerhards [12] evaluated the additional modification of species composition owing to the weed density competition with the investigated crop. To explicate the multifaceted impacts of these edaphic factors on weed data variability, PCA was performed and these diverse soil features were correlated with weed species density. PCA bi-plot analysis signifies the specific composition and distribution patterns of investigated weed species in relation to edaphic factors.

Density and variability of weed species also depend on the inconstancy of both anthropogenic and ecological variables [15]. The essential properties of soil i.e., its pH, fertility, structure, and texture as well as crop rotation, farming practices and availability of moisture strongly impact the weed count and its heterogeneity. Soil analysis of the surveyed fields exhibited that the soil texture varied between sandy clay loam to loam, silty clay loam, silt loam and clay loam (Table 1).

**Table 1:** Physicochemical properties of the soil at 30°C of wheat fields of Sialkot.

Sr No.	Field Name	Texture	pH	TDS	EC	OM	K (ppm)	Na (ppm)	Ca (ppm)	P (ppm)	Zn (ppm)	CaCo_3_ (%)	NaCl (%)	N (%)
**1**	**Chak Mandhaar**	Silty clay loam	8.3±0.05	244±21.2	0.3±0.03	1.4	333.6±5.7	412.3±7.2	0.14±0.01	15±1.1	1.4±0.05	19.3±0.6	1.2±0.06	0.8±0.03
**2**	**Ballanwala**	Silty clay loam	8.3±0.03	229±4.8	0.3±0.02	3.1	438±19.5	458±3.5	0.11±0.002	13.6±1.4	2.2±0.01	18.4±0.3	0.6±0.04	0.8±0.04
**3**	**Saidpur**	Clay loam	8.4±0.01	272±30.3	0.4±0.04	1.4	308.3±4.1	742.6±18.6	0.18±0.008	12.3±1.8	0.8±0.05	18.2±1.1	0.5±0.03	0.7±0.01
**4**	**Kala Khambra**	Sandy clay loam	8.2±0.21	311±37.4	0.4±0.05	1.7	362.6±6.3	660.6±2.4	0.09±0.01	16±1.1	2.3±0.05	14.1±0.6	0.7±0.2	0.8±0.01
**5**	**Pindi Panjoran**	Clay loam	8.3±0.08	222±10.7	0.3±0.02	2.3	379±11.5	526±8.3	0.07±0.006	13.3±2.02	2.3±0.05	15.6±0.3	0.8±0.06	0.55±0.01
**6**	**Lalpur**	Sandy clay loam	8.1±0.33	305±35.3	0.4±0.05	2.4	274.3±8.4	339±3.2	0.17±0.002	12±1.5	2.09±0.02	15.6±0.8	1.03±0.06	0.8±0.01
**7**	**Machi Khokhar**	Sandy clay loam	8.4±0.04	263±32.6	0.4±0.04	1.6	222.3±13.8	226.3±14.1	0.16±0.002	17.3±1.1	1.9±0.03	13.3±1.4	1±0.5	0.7±0.02
**8**	**Kotli Bhutta**	Silt loam	8.2±0.17	234±5.2	0.3±0.01	1.2	155.3±4.7	338±4.5	0.11±0.001	7.7±0.8	4.2±0.08	11.2±0.3	0.5±0.04	0.5±0.01
**9**	**Bhagwal Awanan**	Silty clay loam	8.5±0.06	281±28.4	0.4±0.04	2.6	364.6±4.6	710±7.6	0.18±0.02	17.4±1.7	3.4±0.01	18.5±0.9	0.4±0.03	0.6±0.03
**10**	**Jorian Kalan**	Silty clay loam	8.3±0.12	217±11.2	0.3±0.01	2.1	750±22.6	522.6±6.3	0.13±0.002	19.09±1.04	3.2±0.1	15.3±0.4	0.7±0.1	0.5±0.01
**11**	**Khambranwala**	Loam	8.4±0.01	215±4.6	0.3±0.005	1.65	336.6±26.6	616.6±19.09	0.11±0.001	17.4±0.8	1.1±0.005	7.3±0.4	1.13±0.06	0.8±0.003
**12**	**Ajuwali**	Silt loam	8.5±0.01	241±19.9	0.3±0.03	1.2	332±5.7	418±11.1	0.07±0.001	13.1±0.6	2.2±0.03	14.9±1.07	1.23±0.06	0.5±0.01
**13**	**Salehpur**	Clay loam	8.3±0.003	197±8.2	0.3±0.01	2.1	367.3±8.9	471±3.2	0.19±0.003	4.7±0.7	2.4±0.03	16.6±0.3	1.29±0.01	0.7±0.005
**14**	**Sagarpur**	Silty clay loam	8.3±0.11	203±11.9	0.3±0.01	2.6	301.6±1.2	405±2.8	0.18±0.003	16.9±1.1	2.07±0.01	11.8±0.6	0.6±0.06	0.8±0.01
**15**	**Kapurowaali**	Silty clay loam	8.3±0.02	220±15.2	0.3±0.02	1.6	151.6±13.01	695±3.6	0.13±0.002	10.2±0.3	2.01±0.01	12.1±1.4	0.5±0.01	0.8±0.003

Abbreviations used are TDS (total dissolved solids); OM (organic matter); EC (electrical conductivity).

The estimated soil pH differed from 8.1 to 8.5. EC and TDS ranged from 0.3 to 0.4 mS/cm and 197ppm to 311ppm, respectively. The calcium carbonate %age fluctuated between 6.5 to 20%. NaCl was in the range of 0.0–0.4%, while Nitrogen varied between 0.49 to 0.89%. Meanwhile, the inorganic salts were found as: calcium (0.068ppm to 0.199ppm), sodium (218ppm to 770ppm), phosphorous (3.38ppm to 20.27ppm), potassium (130ppm to 777ppm), and zinc (0.79ppm to 3.44ppm).

Hoveizeh [36] stated that soil properties directly impact weed growth and its distribution. Sperry and Hacke [37] declared that soil texture plays a key role in the maintenance and regulation of infiltration rate and water holding capacity of the soil. Various other investigations also revealed the significance of soil texture and its properties in molding vegetation structure. Passioura [38] demonstrated that the spatial arrangement of soil particles, aggregates and pores is a primary variable that governs vegetation performance. Zhang et al., [39] noted that soil topography and organic matter essentially influence weed composition patterns. It is also hypothesized that soil texture may control nutrient and water availability. Normally, fine-textured soils are rich in organic matter and thus have a greater number of nutrients than coarse-textured soils. Whereas, precipitation percolates to a greater extent through coarse-textured soils in contrast to fine-textured soils [26, 40, 41]. The culmination of current research also acknowledges that divergence of weed species composition was greatly spatially assembled due to specific soil type and its properties.

The present research also correlated various weed species of the wheat fields in Sialkot with each other and various edaphic factors via Pearson’s correlation. Most of these weed species associations were positive. Therefore, the competition and interference between these positively correlated weed species were fairly insignificant. Zhang et al., [42] also demonstrated the succession of weed communities in the rice fields in Pearl River Delta, China, via Spearman rank correlation, Pearson correlation, and point correlation. The current results were in alignment with his work which also indicated that most of the weed species/families showed positive correlation with each other.

In the present study, it was also observed that soil pH was negatively correlated with *C*. *asiatica*, *C*. *album*, and *S*. *oleraceus*. Similarly, *Malva neglecta* showed negative correlation with available nitrogen. A negative relationship was also found among sodium, *C*. *sativa* and *D*. *sanguinallis*. Phosphorous correlated negatively with *A*. *arvensis*, *E*. *helioscopia*, *M*. *denticulata* and *M*. *alba*. Also, weed species including *C*. *dactylon* and *M*. *indicus* showed a negative correlation with soil TDS and calcium carbonate content. The aforementioned results depict that various edaphic factor including soil pH, TDS, nitrogen, CaCo_3_, and inorganic salts (Na and P) substantially influenced weed growth and composition in the investigated wheat fields of Sialkot, Pakistan. Schuster and Diekmann [43] and Stevens et al., [14] also found that pH harms species density whereas, the weed species dominating the USC and UPA correlated positively with clay content, phosphorous and potassium. In inter-correlation of edaphic factors, only EC and TDS were appeared to be having positive correlation with each other. Mostly, the edaphic factors in this study did not show any specific agreement in their existence. This was inconsistence with previous studies as most edaphic factors remained unresponsive to themselves and certain climatic factors such as in Madagascar [44].

Plant species diversity can be commendably estimated using species richness and evenness, however, it is not necessarily true that these components have some relation with each other [41, 45, 46]. But, taking into consideration richness or evenness alone is not a true measure of species diversity. In conformity with previous studies, our sites also varied for their species richness and evenness [47, 48]. However, species richness, and α-diversity were highest at the same sites which are usually the same measure of diversity (S1 Table).

## Conclusions

A quantitative comparison of the prevalent weed species in wheat fields of Sialkot is presented in the current investigation. About 34 weed species associated with 17 families were discovered from 150 quadrats in 15 wheat fields, indicating that the wheat crop of the investigated area is highly susceptible to weed infestation. Most of these weed associations were positive. Also most soil factors were positively correlated with weeds, therefore, the competition and niche separation among these weed species was negligible. However, the edaphic factors significantly influenced the weed density and diversity of the study area. It is also noteworthy that the order of significance of the impact of the evaluated environmental variables is only realistic for the present area of the study and is not an absolute standard. These edaphic variables may act as the vegetation structure determinant in a definite area and a co-factor in others considering the feasible natural resources. The research presents a relevant report to the scientific society regarding the weed flora flourishing in the wheat fields of Sialkot. Thus, the narratives of the current investigation would be valuable in forging a substantial weed management plan as well as in making an insightful discernment in selecting herbicides. However, such survey results from other cereal crops would give a comprehensive picture of the weeds invading the area.

## Supporting information

S1 Table Different diversity indices of weed communities. (DOCX)

S1 Data (XLSX)
